# Structural and Magnetic Response in Bimetallic Core/Shell Magnetic Nanoparticles

**DOI:** 10.3390/nano6040072

**Published:** 2016-04-14

**Authors:** Adeela Nairan, Usman Khan, Munawar Iqbal, Maaz Khan, Khalid Javed, Saira Riaz, Shahzad Naseem, Xiufeng Han

**Affiliations:** 1 Centre for High Energy Physics, University of the Punjab, Lahore 54000, Pakistan; adeela16@gmail.com (A.N.); muniqbal@yahoo.com (M.I.); 2 Institute of Physics, Chinese Academy of Sciences, Beijing 100190, China; xfhan@iphy.ac.cn; 3 Centre for Excellence in Solid State Physics, University of the Punjab, Lahore 54000, Pakistan; saira_cssp@yahoo.com (S.R.); shahzad_naseem@yahoo.com (S.N.); 4 Nanomaterials Research Group, Physics Division PINSTECH, Nilore, Islamabad 45650, Pakistan; maaz@impacs.ac.cn; 5 Department of Physics, Forman Christian College, Lahore 54000, Pakistan; khaliduet@gmail.com

**Keywords:** core/shell nanoparticles, Rietveld refinement, surface effects, FC/ZFC

## Abstract

Bimagnetic monodisperse CoFe_2_O_4_/Fe_3_O_4_ core/shell nanoparticles have been prepared by solution evaporation route. To demonstrate preferential coating of iron oxide onto the surface of ferrite nanoparticles X-ray diffraction (XRD), High resolution transmission electron microscope (HR-TEM) and Raman spectroscopy have been performed. XRD analysis using Rietveld refinement technique confirms single phase nanoparticles with average seed size of about 18 nm and thickness of shell is 3 nm, which corroborates with transmission electron microscopy (TEM) analysis. Low temperature magnetic hysteresis loops showed interesting behavior. We have observed large coercivity 15.8 kOe at *T* = 5 K, whereas maximum saturation magnetization (125 emu/g) is attained at *T* = 100 K for CoFe_2_O_4_/Fe_3_O_4_ core/shell nanoparticles. Saturation magnetization decreases due to structural distortions at the surface of shell below 100 K. Zero field cooled (ZFC) and Field cooled (FC) plots show that synthesized nanoparticles are ferromagnetic till room temperature and it has been noticed that core/shell sample possess high blocking temperature than Cobalt Ferrite. Results indicate that presence of iron oxide shell significantly increases magnetic parameters as compared to the simple cobalt ferrite.

## 1. Introduction

Core/shell (CS) nanostructures with modulated composition and size are an efficient way to construct multicomponent structures that combine various properties of constituent materials in a single system [1,2]. These versatile functional nanomaterials have stimulated great interest due to their novel applications mapping from pure science and technology to biomedical [3,4,5]. Recent advancement has shown continuous increasing interest in bimagnetic CS nanostructure, *i.e.*, where both the core and the shell demonstrate magnetic properties (ferromagnetic/ferrimagnetic and antiferromagnetic). Certainly, for magnetic nanomaterials, CS structure enables the enhancement of and tailoring of magnetic properties such as anisotropy, magnetization reversal process, interparticle interactions, thermal stability of magnetization and coercivity [6]. In fact, exploration of distinct combinations of bimagnetic CS nanomaterials will yield detailed studies on magnetic interaction and exhibit desirable magnetic characteristics for diverse field of applications like permanent magnet, magneto-restrictive devices, magnetic recording, magnetic resonance amplifiers, optimizing hyperthermia and magnetic resonance imaging [7,8]. Furthermore, the advancement in wet chemical synthesis has allowed great control of various parameters like shape, size and composition of nanoparticles, which can also tune the physical and chemical functionalities of these nanomaterials [9,10,11].

In the context of bimagnetic CS nanomaterials, Ferromagnetic/Antiferromagnetic (FM/AFM) or inverse AFM/FM phase structures have been extensively studied [12,13]. Interestingly, in the case of nanoparticles, less attention has been paid to the “exchange spring magnets”, where both hard and soft phases are coupled [14], although it has been reported that, in the case of bulk and thin films, such bimagnetic composites reveal appealing properties [15]. Soft/hard nanocomposite thin films such as Fe_2_O_4_/CoFe_2_O_4_ [16], NiFe/NiCo [17], Fe/CoSm [18], and Fe_3_O_4_/FePt [19] have been prepared through various methods. Studies showed that, in the case of thin films, due to limited interface coupling and reduced homogeneity between both phases, these materials are non-ideal to exploit the numerous enhanced properties. To fulfil the need of maximum exchange interaction between phases, CS nanoparticles would be considered more adequate. These bimagnetic composites can explore properties of both phases like large magnetization and coercivity arising from soft and hard material, respectively [20]. Hard/soft CS nanoparticles of CoFe_2_O_4_/MFe_2_O_4_ (M = Zn, Fe, Mn), Fe/Fe_3_O_4_ [21], FePt/Fe_3_O_4_ [22], and Sm (CoFe)/Fe_3_O_4_ [23] composite materials have been reported, and their results showed enhanced energy product over a single hard phase.

Herein, we present extensive structural and magnetic study of hard/soft CS nanoparticles composed of CoFe_2_O_4_/Fe_3_O_4_ obtained by solution evaporation method. CoFe_2_O_4_ is among one of the most widely used inverse spinel structures due to its novel properties like high thermal, physical and chemically stability, magnetically hard, moderate saturation magnetization and large magneto-crystalline anisotropy field [24]. On the other hand, Fe_3_O_4_ is typically soft ferrite with high saturation magnetization and Curie temperature [25]. The properties of both materials make them appealing for several technological applications like supercapacitors, molecular imaging, spintronics and catalysis.

## 2. Experimental Section

### 2.1. Synthesis of CoFe_2_O_4_ Nanoparticles

The nanoparticles were grown by solution evaporation method. Initially, a solution of 0.1 M Cobalt Nitrate and Iron Nitrate were stirred at room temperature and 0.2 M Oxalic acid was rapidly injected to the solution. In addition, 2 M Nitric acid was added dropwise into the solution to avoid any impurity phases, under vigorous stirring of 30 min. The solution was heated at 120 °C and the heating process was continued until the solution evaporated completely. Afterwards, the obtained product was calcined at 600 °C inside a furnace for 6 h.

### 2.2. Synthesis of CoFe_2_O_4_/Fe_3_O_4_ Core/Shell Magnetic Nanoparticles

For synthesis of CoFe_2_O_4_/Fe_3_O_4_ nanoparticles, 0.2 M Iron Nitrate and Oxalic acid was mixed homogenously and heated at 40 °C for 30 min under constant stirring. Synthesized cobalt ferrite nanoparticles were dispersed in the above solution and were kept under ultrasonic bath for 15 min.

### 2.3. Characterizations

Structural analyses of synthesized nanoparticles were carried out by X-ray diffraction (XRD) (Rigaku D/Max-2400, Beijing, China) and Raman spectroscopy (Horiba JY, Olympus, Beijing, China). XRD was performed by taking a small quantity of powder on an amorphous glass slide using Cu-K_α_ radiation (0.15405 nm). The measurement was carried out in 2θ range of 30°–70° Raman spectra were recorded in the range of 400–900 cm^−1^ at room temperature. Surface morphology was analyzed by transmission electron microscopy (TEM) high resolution-TEM (HR-TEM) (JEOL 2011, Beijing, China), by dispersing the nanoparticles in ethanol and then placing them drop wise onto carbon coated grid. Room temperature and low temperature magnetic measurements of nanoparticles were examined by the physical property measurement system (PPMS) (PPMS-model, 9T, Beijing, China) under applied field of ±5 T.

## 3. Results and Discussion

### 3.1. Structure and Phase Analysis

XRD patterns were obtained to identify structure, phase and crystalline nature of synthesized samples. Figure 1 displays experimental and refined patterns of seed and CS sample annealed at 600 °C. All reflected peaks in Figure 1a,b correspond to the face centered cubic CoFe_2_O_4_ and Fe_3_O_4_ spinel structure. The peaks of CoFe_2_O_4_ and Fe_3_O_4_ are indexed with joint committee on powder diffraction standards (JCPDS) card No.: 22–1086 and 65–3107 respectively. XRD pattern reveals the formation of single phase ferrite structure for both samples without the presence of any impurity phases.

Various structural parameters have been calculated from obtained XRD patterns such as crystallite size, lattice parameter, unit cell volume and X-ray density. Crystallite size has been calculated by using the broadening of the maximum intensity XRD peak (311), appearing around 36.39°. Peak broadening depends on various factors like instrumental effects, strain effect within crystal lattice and finite crystallite size. Scherrer’s formula and the Rietveld refinement method have both been employed to find out crystallite size of the samples. Scherrer’s formula is defined as [26]:

D =δλ/βcosθ

where constant δ depends on the shape of crystallite size (~0.9 for circular shape), λ is the wavelength of used radiation (Cu-K_α_ ~0.1542 nm), β is the full width at half maxima, and θ is Bragg’s diffraction angle. It has been observed that the CS sample has a larger value of crystallite size than the seed nanoparticle by 3 nm. This large value of crystallite size confirms the formation of CS structure.

Laue equation for cubic lattice was used to determine lattice parameter (*a*), defined as [27]:

$$a=d_{hkl}\sqrt{h^{2}+k^{2}+l^{2}}$$

where

$$d_{hkl}=\frac{\lambda }{2\text{sin}\theta }$$

and *d* is interplanar distance and *h*, *k*, *l* are miller indices. Lattice parameter for CoFe_2_O_4_ is in agreement with standard value, whereas lattice parameter of CoFe_2_O_4_/Fe_3_O_4_ is close to the value of the seed nanoparticle. This small difference can be attributed to the lattice mismatch between core and shell, which results in the growth of Fe_3_O_4_ phase on CoFe_2_O_4_ nanoparticles [27,28].

X-ray density of synthesized nanoparticles was calculated by using the following relation [29]:

$$D_{X-\text{ray}}=\frac{8M}{Na^{3}}$$

where *M* is molecular weight of the sample, *N* is Avogadro’s number, and *a*^3^ is unit cell volume. The calculated values show that CS nanoparticles have larger X-ray density as compared to simple core nanoparticles. This increase of *D*_X-ray_ for CS sample is attributed to the increase in molecular weight of the sample. Calculated values of all structural parameters of core (CoFe_2_O_4_) and CS (CoFe_2_O_4_/Fe_3_O_4_) are listed in Table 1.

XRD patterns of both samples were analyzed with the help of Maud software by employing the Rietveld refinement technique using Fd$\bar{3}$m space group [28]. Rietveld refinement is a well established process to explore structural details using powder diffraction data. In the very first step of refinement, background and scale factors were refined. Fitting quality of experimental data is induced by computing goodness of fit (*χ*^2^; which should tend to 1) and two reliability factors—profile factor (*R*_p_) and weighted profile (*R*_wp_; must be close to or less than 10%). The best fit to experimental data is achieved when these factors reach their minimum values. Then, structure is considered as satisfactory.

### 3.2. Raman Spectroscopy

Raman spectroscopy was carried out to get information on structure of synthesized cobalt ferrite and cobalt ferrite/magnetite (core/shell) nanoparticles. CoFe_2_O_4_ has cubic inverse spinel structure with $O_{h}^{7}$(Fd$\bar{3}$m) space group. In this structure, Co^2+^ cations can occupy both octahedral and tetrahedral lattice sites, giving rise to 39 vibrational modes:

A_1g_ + E_g_ + F_1g_ + 3F_2g_ + A_2u_ + 2E_u_ + 4F_1u_ + 2F_2u_

Among these modes, only five are Raman active modes (A_1g_ + E_g_ + 3F_2g_) and four are infrared active (4F_1u_) [30]. Figure 2a represents Raman spectrum for core nanoparticles at room temperature. In this spectrum, the highest frequency mode at 708 cm^−1^ corresponds to the lattice site effects at tetrahedral sites (T-site), while the peak at 472 cm^−1^ reflects lattice site effects in the octahedral site (O-site) [31]. Along with these, the vibrational mode positions 537, 648, 814, and 915 cm^−1^ were also observed in the spectrum.

Figure 2b shows the spectrum of CS nanoparticles. This includes vibrational modes of Fe_3_O_4_ and CoFe_2_O_4_. Like cobalt ferrite, magnetite also has a spinel structure with 56 numbers of atoms per unit cell, containing only 14 atoms in an asymmetric unit, resulting in the presence of 42 vibrational modes in the structure [32];

A_1g_ + E_g_ + T_1g_ + 3T_2g_ + 2A_2u_ + 2E_u_ + 5T_1u_ + 2T_2u_

where only five modes are Raman active vibrational modes (A_1g_ + E_g_ + 3T_2g_), five infrared active (5T_1u_), and the remaining modes (T_1g_ + 2A_2u_ + 2E_u_ + 2T_2u_) are silent in Raman spectra. In the present case, 493, 516, 610, 688 and 698 cm^−1^ modes reflect the presence of Fe_3_O_4_ [33]. However, vibrations around 472, 537, and 814 cm^−1^ show the presence of cobalt ferrite phase in the sample. The Raman study thus showed the formation of single phase core and CS nanoparticles, which is in agreement with XRD observation.

### 3.3. TEM Analysis

Morphology of synthesized CS nanoparticles was investigated by TEM and HR-TEM. In order to avoid aggregation, the product was sonicated in ethanol solution for 20 min before analysis. Obtained micrographs are displayed in Figure 3 where magnetic cores consisting of cobalt ferrite are visible in the dark spots centered by the spherical shell of iron oxide. Figure 3a reports a relatively low magnified TEM image, which shows spherical shaped and reasonably monodispersed CS nanoparticles. Also it can be observed that there is no agglomeration of particles. In Figure 3b, the HR-TEM of core/shell NPs is shown, which illustrates that NPs retain their spherical shape. The core size is in the range of 18 nm with a uniform shell with thickness of about 3 nm.

### 3.4. Magnetic Analysis

To explore magnetic behavior of synthesized nanoparticles, temperature dependence of magnetization (M-T) measured under zero field cooled (ZFC) and field cooled (FC) were carried out with applied field of 1000 Oe. Figure 4a represents FC/ZFC loop for CoFe_2_O_4_ nanoparticles which shows that material is magnetic until room temperature. It can be observed that FC/ZFC curves coincide at high temperature and then diverge significantly from each other as temperature decreases. In a ZFC curve, magnetization increases slowly with increase in temperature and a sharp cusp appeared which corresponds to blocking temperature (*T*_B_), at which thermal energy (*k*_B_*T*) becomes comparable to the magnetic anisotropy energy (*K*_eff_*V*). At blocking temperature, it is considered as [34]:

*K*_eff_*V* = 25 *k*_B_·*T*_B_

where *K*_eff_ is effective anisotropy constant of system, *V* is mean volume of the particle, *k*_B_ is Boltzman constant, and *T*_B_ is blocking temperature. Above *T*_B_, thermal fluctuations become larger than magnetic energy, while below *T*_B_, magnetic energy is larger than thermal fluctuations [35]. In our sample, when *T*_B_ is ~405 K, then FC/ZFC superimpose and bifurcation of both curves occurs, indicating that all nanoparticles are in the same superparamagnetic state.

The observed curves show broadened peak width where the width of the ZFC curve depends on distribution of particle size [36]. If a particle has a particular size, then it would have certain blocking temperature and behave as a ferromagnetic particle, whereas smaller particle size will be attributed to superparamagnetic nature. In our sample, wide peak indicates presence of interparticle/exchange dipole-dipole interactions in the sample.

The FC/ZFC curve for CS nanoparticles is almost similar to the uncoated sample shown in Figure 4b. The divergence of FC/ZFC appears near the maxima of the ZFC curve, which shows that particles are homogeneous in size. However, it can be seen that blocking temperature shifts toward higher temperature. In the case of CS, as the particle size increases, the anisotropy energy also increases which causes a decrease in jump probability across the anisotropy barrier. As a result, blocking temperature transfers toward a high temperature range [37].

M-H loops for core and CS nanoparticles at room and low temperature ranging from 5 to 300 K were obtained from PPMS. Figure 5a shows the hysteresis loops for core nanoparticles, which demonstrate ferrimagnetic nature at all temperatures with interesting magnetic properties. It can be seen from Figure 5a that with a decrease in temperature, magnetic properties such as saturation magnetization and coercivity of sample gradually increases. The reason behind the increase in magnetic properties at low temperature is explained below. The calculated values of Ms and Hc for core nanoparticles are plotted in Figure 6a.

In M-H loop formation of CS nanostructures (Figure 5b), a small kink shape can be seen, which results due to the presence of two mixed magnetic phases (soft and hard) and their exchange interactions [38].

It has been observed that magnetic parameters including remanant magnetization, saturation magnetization and coercivity of CS sample increases remarkably at 5 K. The result shows a significant increase in saturation magnetization values for CS samples as compared to core samples. Initially, saturation magnetization increases monotonically with temperature from 5 to 100 K. The increase in Ms values is considered to be due to the presence of exchange interactions between the magnetic moments of the soft and hard phases. Nevertheless, it is found that magnetization tends to decrease as temperature goes below 100 to 300 K. Such significant decrease in saturation magnetization of CS nanoparticles usually has been attributed to structural distortions at the surface of shell like, spin canting, spin glass and size confinement effects. It has been observed that surface spin disorder can be responsible for exchange anisotropy and existence of spin glass phase around magnetic nanoparticles [39,40].

This spin glass behavior leads to the broken bonds and randomness in exchange interactions on the surface. At low temperature (<100 K), spins of the spin glass layer become aligned and frozen along the applied field. While taking M-H measurements, these spins keep their direction and pin the reversible spins of the core, resulting in the exchange bias effect [41].

Coercivity of CS nanoparticles increases from 1385 to 15844 Oe followed by decrease in ambient temperature, as shown in Figure 6b. Generally, increase in coercivity of magnetic material measures the intrinsic anisotropy of the material [42,43], since, at a particular temperature applied, the field should be enough to overcome any potential barriers and be able to change the orientation of magnetization. Herein, an increase in coercivity can be attributed to the increase in magneto-crystalline anisotropy of the sample combined with strain anisotropy, shape anisotropy, and inter domain coupling [44,45]. This increase in the coercive field also provides evidence for the presence of exchange coupling between soft and hard phases at interface below blocking temperature.

## 4. Conclusions

In conclusion, we have successfully synthesized CoFe_2_O_4_/Fe_3_O_4_ core/shell nanoparticles via the solution evaporation technique. The structural properties have been investigated very carefully and no extra peak was observed in XRD spectra of synthesized samples. XRD patterns indicate the formation of cubic structure for both hard and soft ferrite nanoparticles. Furthermore, Raman spectra also confirm formation of ferrite nanoparticles and the coexistence of both phases (hard and soft) in the case of CS samples. The magnetic measurements confirm the presence of hard/soft structures and exhibit strong exchange interactions between core and shell. It has been observed that magnetic properties increase with a decrease in temperature for CS samples. The results indicate that magnetic properties of hard/soft core-shell nanoparticles can be tuned for specific applications.

## Figures and Tables

**Figure 1:** X-ray diffraction data and Rietveld profile fits of (**a**) core (CoFe_2_O_4_) and (**b**) core/shell (CoFe_2_O_4_/Fe_3_O_4_) ferrite nanoparticles.

**Figure 2:** Room temperature Raman spectra of (**a**) core and (**b**) core/shell ferrite nanoparticles.

**Figure 3:** (**a**) Transmission electron microscopy (TEM) image of core/shell nanoparticles; (**b**) high resolution (HR)-TEM image of core/shell nanoparticles.

**Figure 4:** Temperature dependence of the field cooled (FC) and zero field cooled (ZFC) magnetizations for (**a**) core and (**b**) core/shell ferrite nanoparticles.

**Figure 5:** Magnetization curves recoded at different temperatures ranging from 5 to 300 K for (**a**) core and (**b**) core/shell sample.

**Figure 6:** Variation of the coercivity and saturation magnetization of (**a**) core nanoparticles with temperature and (**b**) core/shell nanoparticles with temperature.

**Table 1:** Structural parameters calculated from X-ray diffraction (XRD) patterns.

Structural Parameters	Core Nanoparticles	Core/Shell Nanoparticles
Crystallite Size (nm)	18.5	21.48
Lattice parameter (Ȧ)	8.177	8.246
Unit cell volume (Ȧ)	546.74	560.69
X-ray density (g/cm^3^)	1.90 × 10^17^	3.79 × 10^17^
